# Biomechanical Process of Skeletal Muscle under Training Condition Based on 3D Visualization Technology

**DOI:** 10.1155/2022/2656405

**Published:** 2022-02-08

**Authors:** Chen Chen

**Affiliations:** Xi'an International Studies University, Xi'an, Shaanxi 710128, China

## Abstract

With the development and popularization of 3D technology, human behavior recognition has gradually developed from plane feature recognition to elevation feature recognition. In the process of collecting motion characteristics, the research on skeletal muscle will lead to a series of data in time series, which is the basis of sports biomechanics research and sports training. Some important semantic information such as centerline and joint center can be obtained by further data processing. The results of the study showed that the three-dimensional coordinate positions of the femur and pelvic attachment points of the muscles surrounding the hip joint from the pelvis were measured and positioned. A 3D model is built to simulate the human skeletal model subjected to speeds of 3 and 7 m/s, and different motion velocities can exhibit different motions. The research in this study shows that using 3D technology and comprehensively utilizing the expertise of biomechanical analysis and graphical modeling to study the mechanical properties of bone joints and soft tissues provide new ways and methods.

## 1. Introduction

The 3D visualization technology of data human body is an important research direction in the field of virtual human modeling. It plays a vital role in the next study of virtual human motion. Biomechanics is an important part of improving athletes' competitive level and training ability [1]. In the three-dimensional finite element analysis of biomechanics, a good three-dimensional finite element model should be first established, and the quality of the model is the first problem and a difficult problem to be solved in the three-dimensional finite element analysis of biomechanics [2]. There are many biomechanical studies on the stress changes in the hip joint, all of which depend on the accurate description of the shape and physiological function of the musculoskeletal system around the skeletal joint [3]. Through biomechanical research on human motion in sports, the main task is to use mathematical methods to mathematically complex systems and then to objectively and quantitatively describe and explain human motion phenomena [4]. In the last few years, because of the development of 3D technology, behavior recognition has begun to make great progress [5–7]. At present, the methods of collecting three-dimensional data from motion can be roughly divided into three categories [8]. One is to mark some locations to capture the action. The second is to reconstruct three-dimensional information from a two-dimensional image sequence [9]. The third method is to use a ranging sensor to describe the motion by distance. The extraction of data on bone and the joint center has become a research hotspot [10]. The extraction of human bones and joint centers based on point cloud data is processed by processing the point cloud data of the real human body acquired by the three-dimensional scanner, thereby extracting semantic information such as the skeleton and joint center of the human body model [11–13].

In this study, we extract the model skeleton through the extraction of 3D structure. The structure not only provides guidance for the segmentation of models but also provides data sources for model skeleton extraction algorithms. Kraft et al. proposed in 1946 that Reeb is used to describe the topology of [14]. Gill et al. used this method to propose the concept of a saddle point for two-dimensional images in 1992 [15]. Pareja-Blanco et al. proposed a series of reference values for the three-dimensional strain of the heart by studying the parameters of normal volunteers [16]. In addition, Thun et al. proposed in 2009 that 3D could establish a complete database in the cycle [17]. Caryn et al. used the joint motion information in-depth video to study human behavior recognition in 2017. This study proposes two methods to recognize human behavior by using the feature vectors representing relative position information and the angle feature vectors representing the angle information [18]. This research direction has also attracted the attention of more and more researchers, and the overall trend of its development has slowly shifted from manual intervention to automated processing [19]. From the attitude-related to the attitude-free transition, the development prospects are very clear. Despite this, the current development status is still not optimistic, and further efforts are needed to achieve an accurate, automatic, fast, and gesture-independent ideal goal of personalized human 3D point cloud data processing [20]. At present, there are still some technical difficulties that need to be solved. The biomechanical study of the myeloid joints is overly biased in mechanics, ignoring anatomical and biological studies [21].

To study the mechanical relationship between the movement of the human internal motor system and the whole-body movement outside the body, this study constitutes the essential grasp of the biomechanical law of human motion behavior and the strain and strain rate imaging technology and technology derived from it is the main technology to detect the strain of skeletal muscle [22]. Each spot can be tracked in successive frames, and the motion trajectory can be calculated so as to accurately track the wall motion and quantitatively analyze it without angle dependence, the continuous passive motion of the knee joint, and computer-aided reinforcement exercise and recovery. The above application examples are enough to prove the unique effects of the simulation technology and database in sports science and medicine [9, 23, 24]. This sophisticated and extensive biomechanical analysis and jingling technology can promote basic research, improve sports equipment, refine athletes' screening/training, and enhance injury prevention and rehabilitation [25]. We hope that regardless of the posture and orientation of the human body during the scanning process, an algorithm can be used to automatically solve the personalized model pose and identify the limbs and torso of the model after acquiring the point cloud data of the model [26]. The model 3D point cloud data obtained by scanning with a noncontact laser scanner is a combination of massive point information and lacks semantic information [27]. In this way, it will inevitably cause certain difficulties in solving the model pose and identifying the model torso and the limbs of the model. If we can get the end feature points of the mannequin, then we can distinguish the torso and limbs of the model by the location of these end feature points. We chose a 3D skeleton-based feature representation method for behavior recognition and used depth typical time warping to align Lie algebra action features [28].

The research of this study shows that it provides a new way and method to study the mechanical properties of bone, joint, and soft tissue by using three-dimensional technology and the professional knowledge of biomechanical analysis and graphical modeling. This study is divided into four parts. The first part introduces the research background that the research of skeletal muscle will produce a series of time series data. In the second part, some important semantic information can be obtained through further data processing. In the third part, a three-dimensional model is established to simulate the human skeleton model with speeds of 3 and 7 m/s. Different motion speeds can show different motions. The results show that it provides a new way and method to study the mechanical properties of bone, joint, and soft tissue by using three-dimensional technology and the professional knowledge of biomechanical analysis and graphical modeling.

## 2. Materials and Methods

In motion, not only musculoskeletal systems need to be simulated, but also these local simulations need to be integrated into the whole human motion for comprehensive analysis. Only in this way can the research results be more complete and practical, and valuable conclusions can be drawn on human health and sports technology. Thus, mechanics and medicine naturally become the two main parts of this subject. The 3D is based on the 2D stereo analysis model of the whole three-dimensional structure, which can more objectively and accurately track the whole trajectory of the myocardium and get the evaluation parameters of rotation, torsion, area change fraction, three-dimensional velocity, and other functions. The finite element method breaks through the limitation of traditional experimental biomechanical research methods and can reconstruct and analyze the structure, shape, load, and mechanical properties of materials that are extremely complex. A new thoracic skeleton mask is generated by region-growing operation, and a preliminary three-dimensional model is constructed. The model is refined by using three-dimensional view mask editing and CT image mask editing functions. In the ankle joint, the foot and the lower leg are at right angles to the normal position. The angle between the lower leg and the back of the foot during exercise is called ankle flexion (buckling), and vice versa. In the normal position, the ankle joint is easily flexed and stretched by the reinforcement of the surrounding ligament. In the movement, the inner edge of the foot is lifted, and the inner side of the foot is turned into the inner turn. Conversely, when the outer edge of the foot is lifted and the sole is turned to the outside, it is called eversion. The surface information of the object can be easily obtained by the 3D scanner. The 3D model of point cloud data based on scanning technology can vividly reproduce the personalized shape information of the human body. It is an accurate and reliable representation method of virtual human geometry. Although a large amount of human body shape information can be provided by this method, this human body shape information does not have human body semantic information. Human body semantic information includes key measurement feature points of the human body, topological structures, and skeletal systems. The coordinate measurement of the muscles around the hip and their attachment points are shown in Table 1 and Figure 1.

The contraction intensity of skeletal muscle is defined as severe, moderate, and mild contraction. The elastic modulus and corresponding muscle strength under three muscle contraction conditions are shown in Table 2 and Figure 2. Elastic modulus is a measure of the resistance of an object to elastic deformation, and the corresponding muscle strength represents the tensile strength of the muscle.

Researchers have made some important achievements in feature extraction, but the current methods still have some shortcomings, such as inaccurate calculation results, low computational efficiency, and the need for tedious manual interaction. There is still a certain distance between practicalities. In depth images, the above problems have been effectively solved, and human contours can be more accurately and effectively extracted. At the same time, this kind of 3D contour can also reflect the motion trajectory of the human side to the camera. At present, many methods based on 3D contour have been proposed. This kind of behavior recognition method based on 3D contour not only uses the information of human body contour itself but also uses histogram and other tools to further reflect the precise information of motion. Each refinement operation depends on the result of the previous operation. The specific process is as follows: in the voxel model, the pixel of a certain point has a certain distribution relationship with its neighboring pixels. According to this feature, certain rules can be drafted to filter it, the redundant information is gradually removed, and the center pixel is retained. It is iterated until there is no redundant information. Although the Achilles tendon is the strongest tendon of the human body, it is rare to have a high level of Achilles tendon rupture. However, it is more common among athletes with short training years, low training levels, or older ages. The reason is that the footwork is irregular or unformed, and sudden intense confrontation causes the Achilles tendon load to be too large and causes breakage. Furthermore, the adductor muscles are divided into two middle and rear muscle units, and the middle and small muscles are divided into three muscle units: front, middle, and back. Although the gluteus maximus is also a relatively wide-ranging muscle, its muscle fibers are parallel and very symmetrical, so they are not further divided. The establishment includes the maxilla (including the tibia and nasal bone), the mandible, the sphenoid bone, the tibia (including part of the parietal bone), the upper dentition, the lower dentition, the temporomandibular joint disc, the joint capsule, the articular cartilage, the joint ligament, the masseter muscle, a three-dimensional finite element model of the diaphragm, pterygoid, and extraptery and complete reduction in the 3D biomechanical environment. The central point of the muscle attachment point is the left pubic symphysis and the right pubic tubercle as measurement points. The measurement process is shown in Table 3 and Figure 3.

The longitudinal strain peaks of the left pubic symphysis and the right pubic tuberosity are shown in Table 4 and Figure 4.

A method of describing motion using 3D skeletal data has gradually attracted widespread attention. This method uses multiple cameras or other sensors to represent the position information of all the joints of each frame in the whole motion by coordinates. The arrangement of the data of each frame in the time series constitutes the whole information of the action. However, there are some shortcomings in skeleton extraction based on topological refinement. For example, the extracted skeleton location is not accurate, the topology structure is complex, limited by three-dimensional space, the amount of data is huge, and the calculation cost is expensive. This makes the method less applied in the field of human body modeling. At the same time, human gravity moves through the foot joints, and the center of gravity alternately moves. It is easy to lose balance. It needs the strong support of the ankle joint, which makes the load of the ankle ligament increase. Additionally, long jump turns are more likely to cause local fatigue of the ankle joint, which can easily cause movement deformation and lead to the occurrence of ankle ligament injury. The method has been gradually applied to many disciplines such as bioengineering and medicine in combination with 3D reconstruction technology and other virtual reality technologies and has become an important experimental method in the field of biomechanics. It can effectively analyze the physical properties of the human body structure, such as the external impact response of the human tissue and the internal stress distribution when subjected to external forces. The speckle-tracking technique based on the high-frame-rate two-dimensional gray-scale image uses the myocardial tissue displayed by the two-dimensional echocardiogram grayscale image as the spot of the innumerable pixel set with the identification feature, and each spot is composed of 10–30 pixels. The material properties of the joint tissues are shown in Table 5 and Figure 5.

Muscle is an important part of the human motion system. Its maximum strength is highly related to muscle shape and depends more on the size of the cross-sectional area of muscle. Therefore, as long as the cross-sectional area of the human muscle is measured, the relative value of muscle strength can be deduced. In various sports, the shape and contraction strength of the original muscle of the hip joint flexion and extension are very important to the successful completion of the special technical movements. A motion vector can be generated by using the position of the template and the matching modes of subsequent frames, and the whole skeletal muscle can be observed by building multiple templates. A circle of triangles around the articular surface of the temporal bone and the neck of the condyle was selected as the common surface, and then, the whole area was selected and deleted to get the upper and lower parts of the articular capsule. The triangle around the articular disc is chosen, and then, the whole area is reverse selected and deleted. The linear model of the periphery of the articular disc requires that the approximate attachment points of the muscles at the proximal and distal ends of the joint are given. It is assumed that the direction of the force transmitted by the muscles accords with the straight-line direction connecting the two points in any case. The central line model requires defining the central line of each muscle and the connection of the central point of each cross section and assumes that the direction of the force transmitted by the muscle at any point is consistent with the tangent direction of the point on the central line. Before dividing the volume mesh into the 3D model, optimization operations are performed such as smoothing and reducing triangles to balance the mesh size and reduce the number of meshes. In this process, multiple parameters are set for quality control, such as maximum geometric error. The angle sets the threshold and the like. After the optimization operation, the model may still have potential problems such as grid inversion and malformation. When the athlete fully stretches to make the toe stand up, the angle of the ankle joint's downward bend increases, and the joint surface force also increases. The stability of the ankle joint is maintained by the talus shape, the connection between the tibia and the tibia. Once a sprain or dislocation occurs, the stability of the ankle joint is bound to decrease. In order to find a suitable correction function in the process of correlation correction of 3D features, we tried different correction functions and selected the best function as our correction function as shown in Table 6 and Figure 6.

Definition of distance transformation proposed in the calibration of human body 3D off-node based on distance transformation is as follows:

(1) $$\begin{array}{c} R_{t}\left(p_{1t},Q_{t}\right)=p_{1t}\cdot \min\left(I_{t}+Q_{t},D_{t}\right)-\left(p_{0t}\cdot Q_{t}+C_{t}\cdot AI_{t}\right)+R_{t-1}. \end{array}$$

The basic idea of the method of directly judging the joint based on the registration image is to register the image as a formula through the image registration algorithm based on the gray difference:

(2) $$\begin{array}{c} I_{t+1}=I_{t}+Q_{t}-\min\left(I_{t}+Q_{t},D_{t}\right)=\max\left(I_{t}+Q_{t}-D_{t},0\right). \end{array}$$

*AI*_*t*_ is a coefficient indicating contrast adjustment, such as a formula:

(3) $$\begin{array}{c} AI_{t}=\frac{\left(I_{t}+Q_{t}\right)+\left(I_{t}+Q_{t}-D_{t}\right)}{2}\\ =I_{t}+Q_{t}-\frac{D_{t}}{2}. \end{array}$$

The calculation formula is determined by using the mean square error criterion in probability statistics:

(4) $$\begin{array}{c} AI_{t}=\frac{\left(I_{t}+Q_{t}\right)}{2}\cdot \frac{\left(I_{t}+Q_{t}\right)}{D_{t}}. \end{array}$$

The critical point is defined, and then, H becomes the critical point of the function:

(5) $$\begin{array}{c} H=\left[h_{1},h_{2},\ldots ,h_{k}\right]=A^{1/2}E. \end{array}$$

An ideal function is used to measure the relationship between points on a three-dimensional human body model:

(6) $$\begin{array}{c} U_{ij}=\frac{H_{ij}}{\sqrt{\sum_{t=1}^{k}H_{it}^{2}}},\;i=1,\ldots ,n,\;j=1,\ldots ,k. \end{array}$$

According to this characteristic, the model end feature points can be defined as follows:

(7) $$\begin{array}{c} \frac{\text{d}x_{1}^{\left(1\right)}}{\text{d}t}+ax_{1}^{\left(1\right)}=\sum_{i=1}^{N}b_{i}x_{i}^{\left(1\right)}, \end{array}$$

where a represents the end feature point of the 3D human body model, and *f* represents the neighborhood of the feature points at the end of the 3D human body model, which can satisfy the following two conditions:

(8) $$\begin{array}{c} \hat{a}={\left(B^{T}B\right)}^{-1}B^{T}Y_{N},\\ f_{\max}^{\prime }=C_{\text{mult}}\cdot f_{\text{avg}}. \end{array}$$

Through the above definition, a conclusion can be drawn that the sum of the geodesic distances between the endpoints of the human body and all the vertices is greater than the sum of the geodesic distances of other points in the neighborhood, and the formula of the number of vertices in the neighborhood is as follows:

(9) $$\begin{array}{c} Dr\left(p\right)=\frac{D\left(p\right)}{\min\left(P_{A},P_{B}\right)},\\ R_{A}\left(p\right)=\frac{\min\left(A_{A},A_{B}\right)}{\max\left(A_{A},A_{B}\right)}. \end{array}$$

A circle is formed by points of the function and connected points. The formula for calculating the level set curve is as follows:

(10) $$\begin{array}{c} \text{Cost}{\left(P\right)}_{i}=\sum_{e\in P_{i}}C\left(e\right). \end{array}$$

Second, according to the formula of the distance between any two points in the space, we can get the following formula:

(11) $$\begin{array}{c} K_{i}=\frac{t*\text{sqrt}\left(Ne\right)+\alpha }{L+\beta }. \end{array}$$

According to the nature of the correlation, the locus of points can be written as follows:

(12) $$\begin{array}{c} G_{g}\left(s\right)=\frac{K_{g}}{1+T_{d0}s}. \end{array}$$

## 3. Result Analysis and Discussion

Bone-based behavior recognition and 3D contour-based behavior recognition have a lot in common. However, compared to the 3D contour behavior recognition method, the bone joint features are not affected by the position of the camera and the appearance of the object. In good bone modeling, the bone-tracking algorithm can acquire joint information from the front, side, or back views so that motion recognition is not affected by the perspective. The traditional method of obtaining human body data is obtained by manually using a measuring tool such as a tape measure, but this method of obtaining human body data is difficult to meet the requirements of accurate, rapid, and large quantities. The 3D point cloud human body data used are obtained through an internationally advanced noncontact laser body scanner, and the in-plane motion is reduced. The articular surface movement is in the knee, and the articular surface motion occurs between the humerus and the femoral condyle and between the femoral condyle and the tibia. Between the humerus and the femoral condyle, the movement simultaneously occurs in all three planes but is minimal on the lateral and frontal planes. Between the femoral condyle and the tibia, the movement simultaneously occurs on one of the frontal and lateral planes. The material properties with the tissue damage limit indicator are introduced into the finite element model, and the damage limit values are directly defined in the bone material attribute assignment process. The finite element software can automatically separate, invalidate, or delete the joints of the skeletal elements, which exceed the damage limit value in the calculation process. In order to display the fracture morphology, the damage morphology is more intuitive, and the damaged skeletal elements are immediately invalidated or deleted in the calculation process. The muscle strength of different muscles is different, and the elastic modulus is different. According to the time taken to complete the displacement, the speed can be calculated. According to the relationship between velocity and strain rate, strain rate can be calculated. Time-based comparisons are shown in Table 7 and Figure 7.

Noncontact 3D scanning technology is the main way to achieve modern human 3D point cloud data acquisition. The acquired 3D point cloud data can be applied to the apparel CAD system so that real human body 3D point cloud data can be used for garment design. The noncontact automatic human body 3D point cloud data acquisition method adopts a photoelectric-based method for acquisition and a laser-based method for acquisition. These two methods of three-dimensional human body scanning technology are based on modern optics, incorporating human body data acquisition technology such as optoelectronics, computer graphics and information processing, and computer vision. The object of behavior recognition is usually a sequence of videos or images in which human motion is discrete, that is, human motion is arranged by a number of stationary skeleton shapes. Therefore, the characterization of human behavior recognition based on 3D bones is to find a way to describe the shape of a static bone. In the learning and control of motor skills, the neuromuscular system achieves the balance and adaptation of external torque and passive reaction torque through the adjustment and control of muscle contraction torque, thereby completing or developing purposeful, efficient, and coordinated human movements. However, in vivo measurement of single muscle force or muscle torque is not possible. Without solving this problem, sports biomechanics is far from guiding sports practice, especially evaluating and guiding muscle strength training. The strain concentration at the corresponding position conforms to the biomechanical response of ribs under direct and indirect external forces. The strain distribution time histograms at different locations of ribs show that the maximum effective strain of the striking rib is similar to that of the posterior rib, but there are many difficulties in establishing the strain distribution time histogram, so it is seldom used at present. In contrast, the linear model is simple, easy to understand, and easy to establish and apply. The data of the medial epicondyle and the external epicondyle of the femur are shown in Table 8 and Figure 8.

The skeleton information in the dataset is processed on the skeleton of the 3D platform output. Due to the nature of 3D, the speed of the video is kept at 20 frames. In the 3D skeleton model, the body parts of the forearm, upper arm, torso, and head are considered rigid bodies. In order to represent each joint, an absolute coordinate system needs to be established. These centerlines can also be called the skeleton of the model. Finally, according to the knowledge of human anatomy, in the vicinity of the human joint, the cross section will have an irregular shape due to the influence of the end of the bone, but the middle part of the bone will have a round shape due to the coverage of the muscle and the contracting tissue. By analyzing the circularity level of the level set curve, the level set curve of the joint center can be determined, and the position of the center of the model joint can be obtained by obtaining the center of gravity of the level set curve. The data smoothing, center of gravity measurement, and velocity parameter formats discussed in the previous hotspots have been completed by standardized software. At present, the development of the graph number analysis method is the function of automatic recognition of human joint points, but this technology relying on gray recognition can only be realized in the laboratory. In the field test, especially when the joint is occluded, it can only rely on manual interpretation of joint points. At the same time, the residual scapular images were removed and the sternoclavicular joints were separated by a three-dimensional view mask-editing operation so that the whole thoracic structure could be independently imaged. Compared with the previous two-dimensional model, it makes it closer to the physiological condition and improves the accuracy of reflecting the joint biomechanical environment. In further research, we intend to use this model to indirectly calculate the stress changes with the change in the position of the center of motion of the medullary joint. In addition, the results of finite element analysis show that the stricken ribs bend locally inward at the striking site, and the striking side thorax withstands the impact energy and undergoes obvious overall deformation and displacement. After a certain distance, springback occurs, which accords with the traditional bone biomechanical response law. The velocity vector of the 3D motion vector is shown in Figure 9.

The correlation between muscle strength and shape is also related to sports. For example, the running and kicking of football players have higher requirements for hip flexion. The speed-skating athlete's thigh sliding has a higher requirement for hip extension. The characteristics of this sports program are beneficial to the development of these muscle groups, and the more obvious the muscle strength, the better the correlation between muscle strength and shape. The greater the knee flexion, the greater the force value of the quadriceps muscle, and therefore, the higher the counter-force value of the patellofemoral joint. If the knee joint is in motion, excessive damage due to normal force and repetitive fine damage will result in injury. This is manifested in many aspects of direct injury that will result in knee joint closure injuries. Indirect injury mechanisms include joint dislocation and rotational or transitive torque, such as collateral ligament injury. At the same time, it is also possible to distinguish the limbs by using the site where the end feature points are located. The horizontal set curve adjacent to the left-hand end feature point exists on the left upper limb, and the horizontal set curve adjacent to the right-hand end feature point exists on the right upper limb. The level set curve adjacent to the feature points at the end of the left foot exists on the left lower limb, and the level set curve adjacent to the feature points at the end of the right foot exists on the right lower limb. The method of the 3D contour is suitable for single action recognition, and the effect of simple atomic action is the best. However, in the process of data superposition, background and noise reduce the accuracy of the contour, and there is much missing information when calculating the two-dimensional mapping of 3D information, so the 3D contour method still has many difficulties in recognizing complex actions. On the contrary, it may lead to erroneous conclusions. Statistical analysis combined with the principles of sports biomechanics is only a digital game. Therefore, in the study of sports biomechanics, attention should be paid not only to the combination of statistical analysis and sports biomechanics but also to the combination of group research and case study. In the process of correlation correction for 3D technical characteristics, the function track is shown in Figure 10.

## 4. Conclusions

The processing of 3D human point cloud data and the acquisition of personalized semantic information related to human body models have become hot and difficult points in the research fields of computer vision, pattern recognition, and intelligent human-machine interface. The elastic modulus of the same muscle is not constant but varies with the contraction strength of the muscle. The different muscle strengths of different muscles determine that the elastic modulus is also different. This experiment assumes that there is a linear relationship between the elastic modulus of the muscle and the muscle strength, and the maximum muscle elastic modulus obtained is related to the maximum muscle strength of the diaphragm, mainly considering the conservation of momentum and the law of momentum transfer and the various aspects of the human body. The principle of mutual relations. In short, the technical characteristics of all kinds of movements are based on the corresponding mechanical principles, with certain regularity. Therefore, in the fully extended position of the skeletal joint, it was found that the rubber band representing the external obturator muscle had slight contact with the femoral neck, and the rubber band representing the sartorius muscle had contact with the rubber band representing the rectus femoris muscle. However, this contact is not obvious and does not significantly change the straight direction of these muscles. The 3D technology can study skeletal muscle by changing the biomechanical characteristics of the longitudinal strain.

## Figures and Tables

**Figure 1:** Coordinate measurement of muscles around the hip and their attachment points.

**Figure 2:** Elastic modulus and corresponding muscle strength under three muscle contraction conditions.

**Figure 3:** The left pubic symphysis and the central point of the right pubic symphysis at the point of muscle attachment were measured.

**Figure 4:** Comparison of peak strains in the longitudinal phase of the left pubic symphysis and right pubic tuberosity.

**Figure 5:** Tissue material properties.

**Figure 6:** Modified function and result.

**Figure 7:** Time comparison of experiments.

**Figure 8:** Data comparison between the medial epicondyle and the external epicondyle of the femur.

**Figure 9:** The 3D motion vector.

**Figure 10:** Function trajectory.

**Table 1:** Coordinate measurement of muscles around the hip and their attachment points.

	Pelvic attachment point	Femur attachment point
Waist muscle	2.54	0.61
Pubic muscle	3.51	1.23
Rectus femoris	4.76	2.21

**Table 2:** Elastic modulus and corresponding muscle strength under three muscle contraction conditions.

Muscle contraction strength	Elastic modulus	Muscle strength
Mild	1.851	8.412
Moderate	3.618	22.641
Severe	9.441	40.541

**Table 3:** The left pubic symphysis and the central point of the right pubic symphysis at the point of muscle attachment were measured.

	Measurements	Modulus value
Left pubic tuberosity	3.8	4.5
Right pubic bone nodule	3.9	4.6

**Table 4:** Comparison of peak strains in the longitudinal phase of the left pubic symphysis and right pubic tuberosity.

	Base segment	Middle section
Left pubic tuberosity	3.64 ± 1.39	5.51 ± 3.45
Right pubic bone nodule	4.34 ± 1.66	5.84 ± 3.56

**Table 5:** Tissue material properties.

Tissue material	Modulus of elasticity	Poisson ratio
Articular cartilage	2.31	0.45
Articular disc	33.11	0.82
Joint capsule	1.11	0.42

**Table 6:** Modified function and result.

Experiment	Function	Result
LARP + DTW	0.90	0.10
LARP + DCTW	0.92	0.11

**Table 7:** Time comparison of experiments.

Experiment	Time (s)	Alignment and classification time (s)
LARP + DTW	623	2520
LARP + DCTW	633	1899

**Table 8:** Data comparison between the medial epicondyle and the external epicondyle of the femur.

	Mean value	Standard deviation
Medial epicondyle of femur	3.55	4.31
Lateral epicondyle of femur	5.21	5.65

## Data Availability

The data used to support the findings of this study are included within the article.
